# Management and Plan of Undergraduates' Mental Health Based on Keyword Extraction

**DOI:** 10.1155/2021/3361755

**Published:** 2021-10-28

**Authors:** Weifeng Zhang

**Affiliations:** Xinxiang University, Xinxiang, Henan 453003, China

## Abstract

Mental health issues are alarmingly on the rise among undergraduates, which have gradually become the focus of social attention. With the emergence of some abnormal events such as more and more undergraduates' suspension, and even suicide due to mental health issues, the social attention to undergraduates' mental health has reached a climax. According to the questionnaire of undergraduates' mental health issues, this paper uses keyword extraction to analyze the management and plan of undergraduates' mental health. Based on the classical TextRank algorithm, this paper proposes an improved TextRank algorithm based on upper approximation rough data-deduction. The experimental results show that the accurate rate, recall rate, and *F*1 of proposed algorithm have been significantly improved, and the experimental results also demonstrate that the proposed algorithm has good performance in running time and physical memory occupation.

## 1. Introduction

The mental health and wellbeing of undergraduates have deteriorated over the last decade. Before the COVID-19 pandemic, higher education was facing a “mental health crisis” [1, 2]. The rapid onset of the COVID-19 pandemic has introduced countless additional stressors, and faculty concern over student wellbeing has increased. Over the past ten or twenty years, the depression has increased from about 25% of undergraduates in 2010 to almost 30% of undergraduates in 2020, and the anxiety of undergraduates has increased from 22% in 2014 to 31% in 2020. Suicidal ideation of undergraduates has increased from 6% in 2010 to 11% in 2020 [3]. The frequency of mental health management organization in undergraduates varies from university to university. Definitely influence of the pandemic on mental health concerns within undergraduates is a big concern. The pandemic has affected the economic development of many countries, and the cooperation of relevant countries on the pandemic has also led to conflicts. The widespread public reports on the Internet and the media have made simple and inexperienced undergraduates unable to distinguish. So, the management and plan of undergraduates' mental health are important under COVID-19 pandemic [4, 5].

Keywords are words that express the central content of a document. Keywords from a document can accurately describe the document's content and facilitate fast information processing. There are two main types of keyword extraction algorithms, which are unsupervised keyword extraction method and supervised keyword extraction method [6–8]. Unsupervised keyword extraction method does not need manually labeled corpus, but it uses some methods to find important words in the text as keywords for keyword extraction. In unsupervised keyword extraction method, candidate words are firstly extracted, and then each candidate word is scored, so top-K candidate words with the highest score are output as keywords. According to different ranking strategies, there are different algorithms such as term frequency-inverse document frequency (TF-IDF), TextRank, and latent Dirichlet allocation (LDA). The supervised keyword extraction method regards the keyword extraction process as a binary classification problem. At first, the candidate words are extracted, and then each candidate word is labeled, so the keyword extraction classifier is trained. When a new document is coming, all candidate words are extracted, and then the trained keyword extraction classifier is used to classify each candidate word. Finally, the candidate words labeled as keywords are used as keywords [9, 10].

Accordingly, the main contributions of this paper are summarized as follows. (i) I study the TextRank keyword extraction algorithm. (ii) An improved TextRank algorithm based on upper approximation rough data-deduction is proposed.

The rest of this paper is structured as follows.  Section 2 reviews the related work. In Section 3, I propose an improved TextRank algorithm based on upper approximation rough data-deduction. The experimental results are shown in Section 4.  Section 5 concludes this paper.

## 2. Related Work

Many strategies of management and plan for undergraduates' mental health have been proposed. In [11], the authors studied to examine student perspectives about college mental health including the primary mental health issues affecting students, common college student stressors, student awareness of campus mental health resources, and mental health topics students wanted more information about. Little research existed into the trends associated with on-campus service utilization for mental health concerns of college students. Rates of broad service utilization existed, but no published study had examined the direct relationship between a range of common mental health symptoms and on-campus service utilization. In [12], the authors studied to explore which common mental health concerns were associated with specific on-campus service utilization in undergraduate students and whether endorsement of more mental health concerns would predict a higher number of services utilized. In [13], the study investigated the moderating role of perceived social support in the relationship between academic demands (measured as perceived academic stress) and mental health of undergraduate students in full-time employment. A growing number of developing countries had experienced worsening air pollution, which had been shown to cause significant health problems. However, few studies had explored the impact of air pollution on the mental health of university students, particularly in the Chinese context. In order to address this gap, in [14], through a large-scale cross-sectional survey, the study aimed to examine the effects of air pollution on final-year Chinese university undergraduates' mental health by employing multivariable logistic regression.

The TextRank algorithm plays an important role in keyword extraction. In [15], the author presented an automatic keyword extraction algorithm based primarily on a weighted TextRank model. In the model, word embedding vectors were used to compute a similarity measure as an edge weight. As a typical keyword extraction technology, TextRank had been used in a wide variety of commercial applications, including text classification, information retrieval, and clustering. In these applications, the parameters of TextRank, including the cooccurrence window size, iteration number, and decay factor, were set roughly. In [16], the authors conducted an empirical study on TextRank, towards finding optimal parameter settings for keyword extraction. The keyword weight propagation in TextRank focused only on word frequency. To improve the performance of the algorithm, in [17], the authors proposed semantic clustering TextRank, a semantic clustering news keyword extraction algorithm based on TextRank. In [18], the authors introduced a new human-annotated Chinese patent dataset and proposed a sentence-ranking-based term frequency-inverse document frequency algorithm for patent keyword extraction, motivated by the thought of “the keywords were in the key sentences.” In the algorithm, a sentence-ranking model was constructed to filter top-K-s percent sentences from each patent based on a sentence semantic graph and heuristic rules. In [19], the authors introduced a word network whose nodes represented words in a document and defined that any keyword extraction method based on a word network was called as a Word-net method. Then, the authors proposed a new network model which considered the influence of sentences and a new word-sentence method based on the new model. In [20], the authors proposed an ontology and enhanced word embedding-based methodology for automatic keyphrase extraction from geoscience documents.

There are also some other methods for keyword extraction. In [21], an enhancement of the term weighting was proposed particularly in the form of a series of modified term frequency-inverse document frequencies, for improving keyword extraction. In [22], the authors proposed an improved rapid automatic keyword extraction method, which used the word string matching feature in the dictionary method to correspond to the relevant execution action function. In [23], a novel text mining approach based on keyword extraction and topic modeling was introduced to identify key concerns and their dynamics of on-site issues for better decision-making process.

## 3. Improved Algorithm Based on Rough Data-Deduction

TextRank keyword extraction algorithm is a graph-based ranking algorithm, which is derived from Google's PageRank algorithm [24]. TextRank firstly divides the target text into several meaningful words and constructs the candidate word graph and then uses the voting mechanism to rank the candidate words to achieve keyword extraction. The task of keyword extraction is to extract several important words from the target text. TextRank algorithm uses the local correlation between words (i.e., cooccurrence sliding window) to determine the correlation between candidate words and then performs iterative calculation and ranking of candidate keywords. Rough set theory is originally used for text classification to speed up classification and improve accuracy. Rough data-deduction is based on rough set theory, which integrates approximate information from upper approximation concept into data reasoning process. This paper introduces upper approximation-based rough data-deduction to TextRank keyword extraction algorithm, and the extracted keywords are used in undergraduates' mental health management and plan.

In TextRank keyword extraction algorithm, the candidate keywords in the text are the graph model constructed by the cooccurrence correlation, and then the weights of each node are calculated by the average transition probability matrix for many times until convergence. After convergence, words are ranked in descending order according to their weights, and the first *N* words are selected as the extracted keywords. This method is more concise and effective, but it has certain limitations. In [25], the convergent operation utilizes a clustering strategy to group the population into multiple clusters. The use of cooccurrence window only considers the correlation between local words, so some words closely related to a certain keyword may be ignored, but keywords from a document are not just limited to the keywords around the words. When doing text keyword extraction, I should fully consider the words in the text as well as some potentially related words. Words with potential correlation will have an important impact on the whole iterative ranking process, and the potential relation can be discovered by the theory of rough data-deduction. Therefore, this paper proposes an improved TextRank algorithm based on upper approximation rough data-deduction.

Based on the word sense similarity of mental health words, the candidate keywords are divided. As there may be a group of words with similar word sense in a document, the weight of this group of words should be increased to improve the accuracy of extraction results when describing the same important content. TextRank algorithm only considers the word sense themselves and ignores the contribution of words with similar word sense. Therefore, the improved algorithm takes the word sense into account and divides the candidate words by word sense, which can extract keywords more effectively.

The rough data-deduction space *M* = (*U*, *N*, *D*) is introduced to describe the keyword extraction of undergraduates' mental health issue structurally. *U* is the universe of discourse (UOD) and the dataset composed of candidate keywords of undergraduates' mental health. *N* is a set of equivalence relation, and *E* ∈ *N*. If and only if *p* is similar to *q*, then *p*, *q* ∈ *U* and <*p*, *q*>∈*E*. D⊆*U* × *U* is defined as *D* = {<*p*, *q*>|*p*, *q* ∈ *U* and there is a relation between *p* and *q*}.

Assuming that deduction correlation is defined as equation (1) by using rough data-deduction,

(1) $$\begin{array}{c} D=\left\{\langle cw_{1},cw_{4}\rangle ,\langle cw_{2},cw_{6}\rangle ,\langle cw_{3},cw_{6}\rangle ,\langle cw_{6},cw_{5}\rangle \right\}, \end{array}$$

where *cw*_1_–*cw*_6_ are the candidate keywords from the text through word segmentation and filtering, and the deduction correlation is determined by the degree of the association rules, that is, pointwise mutual information (PMI).

At the same time, for equivalence relation *E* ∈ *N*,

(2) $$\begin{array}{c} \frac{U}{E}=\left\{\left\{cw_{1},cw_{2},cw_{3}\right\},\left\{cw_{4},cw_{6}\right\},\left\{cw_{5},cw_{7}\right\}\right\}, \end{array}$$

where the equivalence division is based on the similarity between the candidate words.

In rough data-deduction, for candidate word *cw*_1_, the algorithm obtains *cw*_2_ and *cw*_3_ based on similarity rule and then divides *cw*_1_, *cw*_2_, and *cw*_3_ into one dataset, and *cw*_4_–*cw*_7_ can be similarly divided. Then, *cw*_4_ can be obtained from *cw*_1_ based on the degree of the association rules of PMI, as well as *cw*_5_, *cw*_6_, and *cw*_7_. According to rough data-deduction, for *cw*_1_, [*cw*_1_]_*E*_ = {*cw*_1_, *cw*_2_, *cw*_3_}, and [*cw*_1_−*E*] = {*cw*_4_, *cw*_6_}. *E*^*∗*^ ([*cw*_1_−*E*]) = {*cw*_4_, *cw*_6_}, so *cw*_1_⇒_*E*_*cw*_6_. For candidate word *cw*_6_, [*cw*_6_]_*E*_ = {*cw*_4_, *cw*_6_}, and [*cw*_6_-*E*] = {*cw*_5_}. *E*^*∗*^ ([*cw*_6_−*E*]) = {*cw*_5_, *cw*_7_}, so *cw*_6_⇒_*E*_*cw*_7_. *Cw*_1_ = _*E*_*cw*_7_ can be obtained from *cw*_1_⇒_*E*_*cw*_6_ and *cw*_6_⇒_*E*_*cw*_7_. As described, there is also a potential correlation between *cw*_1_ and *cw*_7_, which can provide a certain contribution rate for calculation. The association between candidate keywords is established by the above rules, and the association weight can be added to the iterative calculation process as contribution rate to improve the accuracy of keyword extraction.

The upper approximation-based rough data-deduction to TextRank keyword extraction algorithm is summarized as follows.

**Step 1 .**

Based on TextRank algorithm, the text related to undergraduates' mental health is preprocessed, which includes clause, word segmentation, and part of speech (POS) tagging, and candidate keywords are obtained.

**Step 2 .**

The candidate keywords are divided into different equivalence classes according to their similarities. This paper is divided based on WordNet and Wikitext. For any two candidate words *cw*_1_ and *cw*_2_, the division rule is defined as follows:

(3) $$\begin{array}{c} \text{s}=\omega_{1}s_{1}+\omega_{2}s_{2}, \end{array}$$

where *s*_1_ and *s*_2_ are the similarities calculated by WordNet and Wikitext, respectively. *ω*_1_ and *ω*_2_ are the two weights assigned to *s*_1_ and *s*_2_, and *ω*_1_ + *ω*_2_ = 1.

Assuming that candidate word *cw*_1_ is distributed in WordNet *WN*, and *cw*_2_ is distributed in Wikitext *WT*, the intersection of *WN* and *WT* is *WW*. The value strategy of *ω*_1_ and *ω*_2_ is summarized as follows:

- When *cw*_1_∈*WW* and *cw*_2_∈*WW*, the similarity to *cw*_1_ and *cw*_2_ is calculated based on *WN* and *WT,* respectively, which are denoted as *s*_1_ and *s*_2_. In this paper, *ω*_1_ = *ω*_2_ = 0.5.
- When *cw*_1_∈*WN* and *cw*_2_∈*WN*, or *cw*_1_∈*WT* and *cw*_2_∈*WT*, *cw*_1_ and *cw*_2_ are calculated as *s*_1_ or *s*_2_ based on *WN* and *WT*, where one of the *ω*_1_ and *ω*_2_ is 1, and the other one is 0.
- When *cw*_1_∈*WN* and *cw*_2_∈*WT*, the synonym set of *cw*_2_ is searched based on *WT*, and then the similarity with *cw*_1_ is calculated based on *WN*, and the maximum value is denoted as *s*_1_. If *cw*_2_ has no synonym in *WT*, then *s*_1_ = 0.2, *ω*_1_ = 1, and *ω*_2_ = 0.
- When *cw*_1_∈*WN* and *cw*_2_∈*WW*, the similarity to *cw*_1_ and *cw*_2_ is calculated based on *WN* and denoted as *s*_1_. Then, the synonym set of *cw*_2_ is searched in *WT*, and then the similarity to *cw*_1_ is calculated based on *WN*, and the maximum value is denoted as *s*_2_. If *cw*_2_ has no synonym in *WT*, then *s*_2_ = *s*_1_, and *ω*_1_>*ω*_2_. In this paper, *ω*_1_ = 0.6, and *ω*_2_ = 0.4.
- When *cw*_1_∈*WT* and *cw*_2_∈*WW*, the similarity to *cw*_1_ and *cw*_2_ is calculated based on *WT* and denoted as *s*_2_. Then, the synonym set of *cw*_1_ is searched in *WT*, and then the similarity to *cw*_2_ is calculated based on *WN*, and the maximum value is denoted as *s*_1_. If *cw*_1_ has no synonym in *WT*, then *s*_1_ = *s*_2_, and *ω*_2_>*ω*_1_. In this paper, *ω*_1_ = 0.4, and *ω*_2_ = 0.6.

Here, the calculation of word similarity based on WordNet is defined as follows:

(4) $$\begin{array}{c} s\left(WW_{1},WW\right)=\sum_{m=1}^{3}\ln\;\delta_{m}\prod_{n=1}^{m}s_{n}\left(WW_{1},WW_{2}\right), \end{array}$$

(5) $$\begin{array}{c} s\left(cw_{1},cw_{2}\right)=\underset{m=1\ldots i,n=1\ldots j}{\max}s\left(WW_{1m},WW_{2n}\right). \end{array}$$

In equation (4), *s*_1_(*WW*_1_, *WW*_2_) is the similarity calculated by the set of independent minimum semantic units. *s*_2_(*WW*_1_, *WW*_2_) is the similarity of feature structure of minimal semantic unit of correlation. *s*_3_(*WW*_1_, *WW*_2_) is the similarity of the characteristic structure of the relational sign. The parameter *δ*_*m*_ (1 ≤ *m* ≤ 3) is adjustable and meets the requirement of *δ*_*1*_ + *δ*_*2*_ + *δ*_*3*_ = 1. In this paper, *δ*_*1*_, *δ*_*2*_, and *δ*_*3*_ are set as 0.6, 0.25, and 0.15, respectively. Equation (5) can obtain the sense similarity. When there are multiple senses in a word, equation (5) is used to calculate the maximum similarity among all combinations of senses, that is, the similarity to two words, where *i* is the sense number of the word *cw*_1_, and *j* is the sense number of the word *cw*_2_.

The calculation of word similarity based on *WT* is defined as follows:

(6) $$\begin{array}{c} s\left(WW_{1},WW_{2}\right)=\left(1-0.5dt\left(WW_{1},WW_{2}\right)\right)\sqrt{e^{-di/2j}}, \end{array}$$

where *dt*(*WW*_1_, *WW*_2_) is the distance function of word codes *WW*_1_ and *WW*_2_ in the tree structure. *j* is the total number of nodes in the branch layer, which indicates the number of direct child nodes of the nearest common parent node of two words. *di* represents the distance between branches where two words are located in the nearest public parent node.

**Step 3 .**

The correlation of association rules in rough data-deduction is defined as follows:

(7) $$\begin{array}{c} \mathrm{PMI}\left(cw_{1},cw_{2}\right)=\frac{p\left(CW_{1},CW_{2}\right)}{p\left(CW_{1}\right)p\left(CW_{2}\right)}, \end{array}$$

where *cw*_1_ and *cw*_2_ are two candidate keywords in the text. *p*(*cw*_1_, *cw*_2_) is the probability of *cw*_1_ and *cw*_2_ appearing in the same sentence. *p*(*cw*_1_) is the probability of occurrence of *cw*_1_, and *p*(*cw*_2_) is the probability of occurrence of *cw*_2_.

According to the correlation, the candidate keywords with direct correlation are determined, when *PMI*(*cw*_1_, *cw*_2_) ≠ 0, there is a direct correlation between *cw*_1_ and *cw*_2_, and *cw*_1_, *cw*_2_ and their correlation degrees are stored in the correlation set. Meanwhile, the rough data-deduction relation *D* can be established according to the correlation degree.

Then, by using the rules of rough data-deduction, I get the correlation between the other candidate keywords in all the different equivalence classes, and these words and their correlation degrees are stored into the correlation set.

**Step 4 .**

According to the correlation set obtained in Step 3, candidate keyword graphs with weights are constructed. Then, according to the equation of TextRank algorithm, the weight of each candidate keyword is calculated iteratively until convergence.

## 4. Experiment and Results Analysis

### 4.1. Experimental Data and Evaluation Criteria

The experiment selects 26300 questionnaires of mental health management of undergraduates from Xinxiang University with 23 schools and 60 majors, which consist of psychological distress, depression, suicidal tendency, and self-evaluation related to mental health within 300 to 1000 words. In particular, these undergraduates are distributed for different grades uniformly. The 19000 valid questionnaires are obtained by excluding questionnaires with self-evaluation less than 300 words to test the effect of proposed method in this paper. The questionnaires use silver ink with a metal oxide [26]. 10 keywords of each questionnaire are extracted and ranked by the importance. In this paper, *ω*_1_ and *ω*_2_ are set 0.5.

In addition, for comparison purposes, TextRank, a keyword extraction using supervised cumulative TextRank (KESCT) [27], scientific research project TF-IDF (SRP-TF-IDF) [28], and high representation tags LDA (HRT-LDA) [29] are selected. Three evaluation indexes commonly used in classification are used to compare and evaluate the quality of experimental results, which include precision (*P*), recall rate (*R*), and *F*1 (*F*). *P* is the accuracy of extraction results. *R* is the coverage degree of the extraction results to the correct keywords. *F* is a comprehensive evaluation index of harmonic average of *P* and *R*.

### 4.2. Experimental Results

It is found in the experiment that the two important parameters can affect the keyword extraction result of TextRank algorithm, which are the cooccurrence window size and the number of keywords, while the implementation of TF-IDF algorithm based on statistical feature and the algorithm proposed in this paper are not affected by the cooccurrence window size. I set the number of extracted keywords as 10, and the value of the comparison window is within [4, 10]. The *F*1 under different cooccurrence window sizes is shown in Figure 1.

It can be seen from Figure 1 that TextRank algorithm has different extraction effects under different cooccurrence window sizes. In the same test set, this paper compares the effect of different cooccurrence window sizes, and when the cooccurrence window size is 5, the original TextRank algorithm has the best extraction effect with high *F* value. Therefore, in order to ensure the effectiveness of the proposed algorithm, the cooccurrence window size is set to 5.

The initial window value is set to 5, and *P*, *R*, and *F* are calculated with the number of keywords within [3, 10]. The calculation results are shown in Table 1.

At the same time, in order to observe the experimental results of five algorithms conveniently, the *P*, *R,* and *F* of the algorithm are plotted, as shown in Figures 2–4.

Figure 2 describes the variation trend of the accuracy of the five algorithms when extracting different numbers of mental health keywords. As can be seen from Figure 2, with the increasing number of mental health keywords extracted, the accuracy of each algorithm decreases, but the accuracy of the algorithm proposed in this paper is always higher than other four baselines. The TextRank algorithm based on rough data-deduction proposed in this paper will integrate upper approximation information into the process of data-deduction so that the mutual deduction between data presents the characteristics of approximate entailment or imprecise association, and the potential association between candidate keywords can be mined. If the potential association is added to the iterative calculation of the weight of each candidate keyword, more accurate extraction results can be obtained. Therefore, the accuracy of the algorithm proposed in this paper is theoretically higher, and its accuracy *P* value is higher than other four baselines.

Figure 3 describes the change of recall rate of five algorithms when extracting different numbers of mental health keywords. In Figure 3, the recall rate of the algorithm proposed in this paper is higher than that of other four baselines, and the recall rate increases with the increasing number of mental health keywords. The SRP-TF-IDF algorithm relies too heavily on word frequency and does not use correlation between words at all. KESCT algorithm adopts the cooccurrence window principle. Although the relation between words is considered, the algorithm is more inclined to put forward frequent words due to its limitations, which may ignore important words with low word frequency that can describe the topics. However, the rough data-deduction used in this paper can expand the correlation range and enhance the coverage of the keywords of the correct correlation in order to improve the recall rate of the algorithm. The influence of word frequency decreases with the increasing number of keywords, and the advantages of the algorithm proposed in this paper will be more obvious.

Figure 4 describes the *F* values of five algorithms when extracting different numbers of mental health keywords. When evaluating the experimental results, it is expected that both *P* and *R* should be as high as possible. However, in most cases, the two values are contradictory. Therefore, *F* value should be used to comprehensively consider the two values, which can reflect the effectiveness of the whole algorithm. Keyword extraction based on rough data-deduction can mine the potential association between candidate keywords theoretically, which increases the candidate words and range of the association. The keyword extraction based on rough data-deduction adds the potential association to the iterative calculation of the weight of each candidate keyword, so the extraction results will be more accurate, that is, the algorithm is also more effective.

According to the experimental results, the proposed algorithm has higher *P* and *R* than the other four baselines. The *F* will be higher with the higher *P* and *R*, and the higher *F* can indicate the effectiveness of the algorithm. In conclusion, the accuracy rate, recall rate, and comprehensive evaluation index *F*1 of the proposed algorithm are higher than those of the four baselines, which indicates that the improved TextRank algorithm based on upper approximation rough data-deduction is more effective in mental health keyword extraction.

The test set of this paper uses the self-evaluation in the questionnaire of undergraduates' mental health. The text length is generally less than 500 words, which is mainly concentrated in 300–500 words. This paper divides the test set by the number of self-evaluation words. Each test set randomly selects 30 texts of corresponding text words to compare the running time and physical memory occupation of the five algorithms.

As can be seen from Figure 5, when the number of words in the text is 300–400, the number of deduction and semantic calculation is small, and the running time of the algorithm is also short. The number of deduction and semantic calculations increases with the increasing number of words. Compared with TextRank, the running time of the proposed method is still shorter than that of the other three baselines, which is similar to TextRank's efficiency.

It can be seen from Figure 6 that the physical memory occupation of the proposed method is small with good efficiency. When the number of words in the text is 600–800 or 800–1000, the physical memory occupation of SRP-TF-IDF and KESCT is nearly the same.

This paper manages the undergraduates' mental health through the keyword extraction. The results show that academic problem, emotional problem, interpersonal problem, anxiety problem, sexual problem, and adaptation to college life are the universal mental health issues of undergraduates. Currently, how to deal with mental crisis is an urgent problem that colleges cannot avoid. The proposed bounded area elimination algorithm in [30] analyzes the feature extraction, and the idea of feature extraction is similar to the TextRank keyword extraction algorithm proposed in this paper . Timely plan of mental health crisis is to provide supports and help to those who have experienced personal crisis so that they can restore their mental balance and have full confidence in life.

## 5. Conclusions

In a fast-paced society, there is more competition among undergraduates, that is, they are facing the dual pressure of enrollment and employment, and mental health is very important for them. Mental health is the necessary condition and foundation for everyone's all-round development in today's society, which is also a necessary psychological quality for undergraduates. This paper introduces upper approximation-based rough data-deduction to TextRank keyword extraction algorithm, and the extracted keywords are used in undergraduates' mental health management and plan. The comparison experiments reveal that the proposed algorithm outperforms four baselines in terms of accuracy rate, recall rate, *F*1, running time, and physical memory occupation.

The future works are stated as follows. (i) The deduction rules of rough data will be further refined and improved, so as to get better extraction effect. (ii) The words related to mental health may be incomplete in WordNet and Wikitext, which results in unsatisfactory keyword extraction. The following research will consider using a corpus of mental health related to achieve keyword extraction.

## Figures and Tables

**Figure 1:** *F* value under different cooccurrence window sizes.

**Figure 2:** The comparison of *P* of the five algorithms.

**Figure 3:** The comparison of *R* of the five algorithms.

**Figure 4:** The comparison of *F* of the five algorithms.

**Figure 5:** The comparison of running time of keyword extraction algorithms.

**Figure 6:** The comparison of physical memory occupation of keyword extraction algorithms.

**Table 1:** The comparison of experimental results of five algorithms.

The number of keywords	Algorithm	*P* (%)	*R* (%)	*F* (%)
3	TextRank	52.32	15.50	23.79
	KESCT	55.03	22.35	30.08
	SRP-TF-IDF	64.10	23.00	33.59
	HRT-LDA	70.54	24.56	34.16
	This paper	80.67	29.30	36.51
4	TextRank	49.06	19.71	28.01
	KESCT	54.76	24.33	33.08
	SRP-TF-IDF	62.15	26.94	34.15
	HRT-LDA	69.87	29.41	35.09
	This paper	79.06	31.08	43.66
5	TextRank	48.51	25.16	32.18
	KESCT	52.61	27.66	36.07
	SRP-TF-IDF	60.48	28.54	37.22
	HRT-LDA	66.92	30.69	39.05
	This paper	78.35	32.17	47.65
6	TextRank	42.67	27.65	32.01
	KESCT	49.62	30.25	36.95
	SRP-TF-IDF	55.40	32.49	34.12
	HRT-LDA	60.73	34.16	40.08
	This paper	77.70	39.58	51.89
7	TextRank	41.19	29.90	33.77
	KESCT	45.12	34.15	33.99
	SRP-TF-IDF	50.08	36.58	40.06
	HRT-LDA	55.64	38.04	45.37
	This paper	74.39	45.89	54.68
8	TextRank	39.66	31.57	34.55
	KESCT	40.51	35.26	32.89
	SRP-TF-IDF	45.99	38.16	39.98
	HRT-LDA	49.30	42.53	44.38
	This paper	70.88	50.07	55.81
9	TextRank	36.78	32.36	33.99
	KESCT	37.41	36.45	34.01
	SRP-TF-IDF	44.01	40.19	40.71
	HRT-LDA	40.09	45.20	46.39
	This paper	65.72	55.06	56.09
10	TextRank	35.87	35.64	33.87
	KESCT	33.02	40.16	33.66
	SRP-TF-IDF	38.28	42.26	38.74
	HRT-LDA	39.16	49.39	43.91
	This paper	60.10	59.03	55.99

## Data Availability

All data used to support the findings of the study are included within the article.
